# Image Mosaic Algorithm-Based Analysis of Pathological Characteristics of Gastric Polyp Patients Using Computed Tomography Images

This article has been retracted.

**DOI:** 10.1155/2021/6086106

**Published:** 2021-11-09

**Authors:** Xiqi Zhu, Jian Jiang, Jian Wang, Yue Tang, Xiaoming Ge

**Affiliations:** Department of General Surgery, Wuxi Second People's Hospital, Wuxi 214002, Jiangsu, China

## Abstract

The application value of image mosaic algorithm (IMA) based CT imaging technology in the analysis of pathological characteristics of gastric polyp (GP) patients was explored in this work. 588 cases of GP patients in the hospital were selected as the research objects, and CT images based on IMA were adopted for examination. The patient's basic information, image performance, and gastroscopy results were recorded. The results showed that the absolute mean bright error (AMBE) index and information entropy of the IMA are 0.0625 and 7.0385, respectively. The clinical symptoms of patients were mostly abdominal pain (21.4%), abdominal distension (15.6%), and sour regurgitation (17.8%). The common size of GP was no more than 0.5 cm, and the common type was Yamada type II. There were notable differences between single and multiple GPs of different pathological types (*P* < 0.05). Proliferative polyps were mostly found in the stomach and antrum, while fundus gland polyps were mostly in the stomach and fundus. There was significant difference between the growth location of the hyperplastic polyp and basal gland polyp (*P* < 0.05). In summary, the CT images of IMA proposed in this paper can not only realize image splicing effectively but also were superior to the traditional SIFT method in the quality of splicing image and were conducive to the analysis of the pathological characteristics of GP patients, which had significant clinical promotion value.

## 1. Introduction

Gastric polyp (GP) is a raised lesion caused by gastric mucosal epithelium or submucosa with pedicle or sessile and protrudes into the gastric cavity [1, 2]. It is usually regarded as a benign tumor of gastric epithelium or gastric interstitial origin. With the improvement of living standards of people, the occurrence of GP is getting higher and higher. However, the cause and mechanism of GP are still unclear. Studies have shown that the occurrence of GP may be related to environment, diet, genetic factors, and *Helicobacter pylori* (HP) infection [3]. The potential for malignant transformation of adenomatous polyps is extremely high. Some scholars also found that malignant transformation also existed in hyperplastic polyps. GP is usually found when the patient is undergoing endoscopy, and the clinical symptoms of the patient are mainly stomach pain, abdominal pain, and indigestion [4, 5]. Since GP is not specific in clinical manifestations and is similar to gastric tumors, it is easily misdiagnosed, so early diagnosis is more difficult. How to adopt effective diagnostic methods to distinguish GP from early gastric cancer and gastric schwannoma is of great significance for the early prevention and subsequent treatment of GP.

Clinically, the examination methods for GP are mainly endoscopy, ultrasound, and CT imaging [6, 7]. Endoscopy is performed by inserting through mouth into the stomach to intuitively understand the gastric lesions, but the examination process may cause discomfort for patients. Ultrasonography has a high diagnostic value for gastric diseases, especially for gastric cancer with obvious mass. However, ultrasonography cannot produce a significant contrast for gastric ulcers and gastric polyps with low echo. CT imaging technology has advantages such as noninvasiveness, and its advantages are more significant. CT imaging technology can clearly and intuitively present tumor morphological characteristics, location distribution, size, edge, and other information as well as understand the internal structure of the tumor and its relationship with surrounding tissues, which is widely utilized in the clinical diagnosis of gastric diseases [8]. With the increasing application of CT technology in the medical field, the medical image mosaic method has become a hot and difficult spot in medical image processing. Image mosaic technology is a novel image technology that adopts the computer to match and align overlapping images and finally synthesize complete image information [9, 10]. Image mosaic usually includes image acquisition, image registration, and image synthesis, among which, image registration is the key to image mosaic. The obtained images cannot be of simultaneously high resolution and high matching. Scale-invariant feature transform (SIFT) algorithm is a common feature extraction and matching algorithm, which has ideal matching characteristics and stability in image scaling and rotation transformation [11]. SIFT is currently a hotspot in image matching, and many stitching algorithms are based on the SIFT algorithm. Based on the above advantages, SIFT feature vectors were fused with image regional feature vectors, and new feature vectors were constructed for feature point matching to complete medical image registration and stitching. CT imaging technology based on IMA was proposed and applied to the analysis of pathological characteristics of GP patients, to provide a theoretical basis for the clinical diagnosis and follow-up treatment of GP diseases.

## 2. Materials and Methods

### 2.1. Research Objects and Grouping

588 GP patients admitted to the hospital from October 2016 to July 2020 were selected as study objects, including 154 males and 434 females, ranging in age from 20 to 88 years old, with an average age of 58.98 ± 9.37 years old. This experiment had been approved by the ethics committee of the hospital, and all the patients included in the study had known about the treatment and agreed to it.

Inclusion criteria: (1) patients had completed the histopathological diagnosis; (2) patients had no contraindications for gastroscopy; (3) patients with all parts inspected carefully and the process was complete; and (4) patients with complete clinical data. Exclusion criteria: (1) patients underwent gastric surgery; (2) patients with inflammatory bowel disease; (3) patients with gastric cancer, familial adenomatous polyposis (FAP), or juvenile polyposis (JPS); and (4) patients with incomplete clinical data.

### 2.2. CT Examination Method

Imaging diagnosis was performed with a Sensation 64-slice spiral CT scanner (Siemens, Germany). The patient fasted for 4 h before examination, drank 100 mL water 30 minutes before the examination, and drank 300–500 mL again during examination. The patients' stomach and duodenum were fully inflated and performed under the condition of holding their breath. The scan site is the stomach fundus cardia and gastric antrum. The scanning parameters were set as follows: a layer thickness of 3 mm for continuous uninterrupted scanning with 120 kV and 200 mAs scanning voltage. Omnipague contrast agent was utilized to inject about 300 mgI/mL from the patient's anterior cubital vein at a rate of about 3.5 mL/s and a dose of 2 mL/kg.

### 2.3. CT Image Based on Image Mosaic Algorithm

Image stitching technology generally includes image preprocessing, image registration, and image synthesis. The flow of IMA is shown in Figure 1. Medical image preprocessing mainly removes noise in CT images and enhances the images. Then, the SIFT algorithm is utilized to find the corresponding points of the two CT images, and the initial corresponding point set is obtained. After that, the statistical slope maximum method and the random sample consensus (RANSAC) algorithm are adopted to eliminate the mismatch, and the final corresponding point set is obtained. Finally, the two obtained CT images are stitched to obtain the stitched image.

SIFT algorithm performs feature extraction on CT images, and the scale space image of the image can be represented as follows.

(1) $$\begin{array}{c} L\left(x,y,\sigma \right)=A\left(x,y\right)⊗G\left(x,y,\sigma \right). \end{array}$$

Here, *G*(*x*, *y*, *σ*) is the Gaussian function; *L*(*x*, *y*, *σ*) is the scale space image; and ⊗ is the convolution symbol.

Difference of Gaussian scale-space (DOG) is adopted to detect the stability of feature points.

(2) $$\begin{array}{c} D\left(x,y,\sigma \right)=\left(G\left(x,y,k\sigma \right)-G\left(x,y,\sigma \right)\right)⊗A\left(x,y\right),\\ =A\left(x,y,k\sigma \right)-A\left(x,y,\sigma \right). \end{array}$$

(3) $$\begin{array}{c} \frac{\partial G}{\partial \sigma }=\sigma \nabla^{2}G,\\ \frac{\partial G}{\partial \sigma }\approx \frac{G\left(x,y,k\sigma \right)-G\left(x,y,\sigma \right)}{k\sigma -\sigma }. \end{array}$$

Based on equation (3), the following equation can be acquired:

(4) $$\begin{array}{c} G\left(x,y,k\sigma \right)-G\left(x,y,\sigma \right)=\left(k-1\right)\sigma^{2}\nabla^{2}G. \end{array}$$

Equation (4) can approximately represent the DOG image, and then the image is selected to determine the extremum. The extremum points are marked as candidate points, and the Taylor formula is adopted to perform the following calculations:

(5) $$\begin{array}{c} D\left(x\right)=D+\frac{\partial D}{\partial x}x+\frac{1}{2}x^{T}\frac{\partial^{2}D}{\partial x^{2}}x. \end{array}$$

In equation (5), *x*=(*x*, *y*, *σ*) is the coordinate of the candidate point; *D* is the DOG image value of the candidate point; and 1/2*x*^*T*^∂^2^*D*/∂*x*^2^*x* is close to zero.

The exact position of the extreme point is obtained as follows:

(6) $$\begin{array}{c} x=-\frac{\partial D}{\partial x}{\left(\frac{\partial^{2}D}{\partial x^{2}}\right)}^{-1}. \end{array}$$

The gradient magnitude *m* and gradient direction *θ* of the feature point are expressed as follows:

(7) $$\begin{array}{c} m\left(x,y\right)=\sqrt{\left(L\left(x+1,y\right)-L{\left(x-1,y\right)}^{2}+\left(L\left(x,y+1\right)-L{\left(x,y-1\right)}^{2}\right)\right.}\\ \theta \left(x,y\right)=\arctan\;t\left(\frac{\left(L\left(x,y+1\right)-L\left(x,y-1\right)\right)}{\left(L\left(x+1,y\right)-L\left(x-1,y\right)\right)}\right). \end{array}$$

The coordinate axis is rotated to the main direction of the feature point, and the 8 × 8 neighborhood is selected. The size and direction of the gradient after the rotation operation are calculated, and then Gaussian window smoothing is carried out. It is divided into four regions, eight directional gradient histograms in the four regions are counted, and then the feature vectors of feature points are obtained. For the feature vectors obtained by the SIFT algorithm, the similarity measure is adopted to measure the similarity of regional feature vectors, and the calculation is as follows:

(8) $$\begin{array}{c} \chi^{2}=\frac{1}{2}\sum_{K}\frac{{\left(SC_{i,k}-SC_{j,k}\right)}^{2}}{SC_{i,k}-SC_{j,k}}. \end{array}$$

At the same time, the threshold value *T* is set. If the similarity measure is less than *T*, the corresponding points are paired correctly.

For the paired feature points, (*x*_*i*_, *y*_*i*_) is projected to the reference plane through the transformation matrix and then projected to the plane where (*x*_*j*_, *y*_*j*_) is, and the distance difference is as follows:

(9) $$\begin{array}{c} d_{ij}=\sqrt{{\left(x_{j}-x_{i}^{\prime }\right)}^{2}+{\left(y_{j}-y_{i}^{\prime }\right)}^{2}}. \end{array}$$

The optimization objective function expression (*E*) is as follows:

(10) $$\begin{array}{c} E=\sum f{\left(d_{ij}\right)}^{2}. \end{array}$$

Then, the following equation is obtained:

(11) $$\begin{array}{c} M_{i}=M_{ik}^{\prime }M_{k}. \end{array}$$

In equation (11), *M*_*ik*_′ is the update amount of the transformation matrix, and *M*_*k*_ is the transformation matrix from the best adjacent image to the reference image.

### 2.4. Observation Indexes

The patient's basic personal information, CT image results, and gastroscopy results were recorded. Basic information includes gender, age, smoking, and drinking condition. Gastroscopy included polyp growth site, pathological type, number, and *Helicobacter pylori* (HP) infection. Yamada typing was referred for morphological classification, and HP infection was detected by rapid urease test.

### 2.5. Simulation Experiment Design

The CT image processing results of different image stitching and segmentation algorithms are shown in Figure 2. The information entropy and absolute mean bright error (AMBE) index are taken to evaluate the image mosaic quality. It is assumed that the original image *x* (*i*, *j*) and the processed image *y* (*i*, *j*) have *F M* *×* *N* gray levels, and the gray distribution density of the processed image is as follows:

(12) $$\begin{array}{c} \left\{\begin{array}{c} \rho \left(x\right)=\rho \left\{F=x\right\}x\in F,\\ \text{AMBE}=M\left(X\right)-M\left(Y\right). \end{array}\right. \end{array}$$

The information entropy expression is as follows:

(13) $$\begin{array}{c} H\left(x\right)=-\sum_{x\in L}p\left(x\right)\log_{2}\;p\left(x\right). \end{array}$$

Here, *H* represents information entropy. The expression of AMBE is as follows:

(14) $$\begin{array}{c} \text{AMBE}=M\left(X\right)-M\left(Y\right). \end{array}$$

*M*(*X)* and *M*(*Y)* are the average gray values of the original image and the processed image, respectively. The larger the information entropy value is, the more information in the image is and the higher the image quality is. The larger the AMBE, the larger the average brightness error of the original image and the processed image.

### 2.6. Analysis of CT Images

CT image analysis is mainly to determine the length and short diameter of the largest layer of the tumor and observe the location, size, shape, growth mode of the tumor, whether calcification, cystic changes, uniform, or uneven enhancement. The central location of the largest layer of the tumor was taken to avoid cystic degeneration, calcification area, and bleeding area, and the area of interest was about 0.1–0.25 cm^2^.

### 2.7. Statistical Methods

SPSS20.0 statistical software was adopted for analysis. Measurement data were expressed as mean ± standard deviation ($\bar{x}$ ± *s*), and *t*-test was utilized for comparative analysis; measurement data were expressed as percentage (%), tested by *χ*^2^ test for comparison and analysis between groups. If *P* < 0.05, the difference was statistically significant.

## 3. Results

### 3.1. CT Image Results Based on Image Mosaic Algorithm

The AMBE and information entropy values of the algorithm proposed in this work are 0.0625 and 7.0385, respectively. The traditional SIFT algorithm has insufficient detection speed and matching accuracy of feature points in the process of image registration, so it cannot carry out edge detection and image enhancement preprocessing of medical images before splicing. The image stitching CT image algorithm proposed in this work can not only effectively realize image stitching but also is superior to the traditional SIFT method in terms of stitched image quality.

### 3.2. CT Imaging Characteristics of Gastric Polyp Patient

The results of CT imaging of some patients are shown in Figure 3. Patient A had abdominal distension accompanied with hiccups for half a year. The pathological results showed fundus gland polyps. CT examination showed round soft tissue masses in the fundus of the stomach. Patient B had symptoms of abdominal distension for 1 month. The pathological examination results showed multiple hyperplastic polyps in the antrum. CT examination showed that there were multiple and irregular soft tissue masses in the antrum. The pathological examination result of patient C was hyperplastic polyp in the antrum. CT scan showed a round mass with pedicled soft tissue in the antrum.

### 3.3. General Information of GP Patients

The gender distribution of patients of different age groups and the distribution of the number of patients is shown in Figure 4 and Figure 5, respectively. Figure 4 revealed that there were 10 males and 15 females in patients aged 0–40 years; 17 males and 56 females in patients aged 40–49 years; 35 males and 136 females in patients aged 50–59 years; 57 males and 159 females in patients aged 60–69; and 35 males and 68 females aged over 70 years. There was a total of 588 GP patients, including 154 males and 434 females, and the male to female ratio was 1 : 2.818. The number of females was relatively larger, and their prevalence was higher. Figure 5 shows that the distribution of GP patients was the most in the 60–69 age group (216 people, 36.73%), followed by the 50–59 age group, which accounted for 29.08% (171 cases). There were 25 patients aged 0–40 years old, 73 patients aged 40–49 years old, and 103 patients aged 70 years or older.

The distribution of smoking and drinking of GP patients is shown in Figure 6. The comparisons of different pathological types showed that patients with gastric gland polyps and adenomatous polyps had evident differences in whether they smoked or not (*P* < 0.05), while patients with other pathological types were not comparable regarding the smoking conditions (*P* > 0.05). There was no notable difference among the pathological types regarding whether patients drank alcohol (*P* > 0.05).

### 3.4. Clinical Symptoms of GP Patients

The patient's clinical symptoms are shown in Figure 7. The proportion of patients with abdominal discomfort was 5.5%, retrosternal discomfort patients accounted for 2.2%, weight loss for 2.3%, nausea and vomiting for 5.4%, abdominal pain for 21.4%, abdominal distension for 15.6%, sour regurgitation for 17.8%, and heartburn for 16.2%.

### 3.5. Characteristics of Pathological Types of GP Patients

The distribution of patients with different pathological types is shown in Figure 8. The proportion of patients with inflammatory polyps was 8.76%, adenomatous polyps accounted for 2.03%, chronic inflammation accounted for 3.08%, inflammatory fibrous polyps accounted for 1.26%, fundus gland polyps accounted for 48.25%, and hyperplastic polyps accounted for 36.62%.

Table 1 shows the GP size and Yamada typing results. Polyp sizes of ≤0.5 cm, 0.6–1 cm, 1.1–2 cm, and ≥2 cm accounted for 71.2%, 20.3%, 5.7%, and 2.8%, respectively. The size distribution of polyps of each pathological type was highly comparable (*P* < 0.05). Yamada types I, II, III, and IV patients accounted for 21.1%, 75.3%, 3.3%, and 0.3%, respectively. Types I and II accounted for more, with considerable differences relative to other types (*P* < 0.05).

The distribution of different pathological types of GP is shown in Table 2. GP was present in all parts of the gastric cavity, and the incidence of gastric fundus and gastric body was relatively higher, accounting for 28.62% and 36.85%, respectively. The pairwise comparison of different pathological types of polyps revealed that proliferative polyps were mostly found in the stomach and antrum, and fundus gland polyps were mostly found in the stomach and fundus. The growth position between the two groups was considerable (*P* < 0.05), but there was no evident difference between the other types (*P* > 0.05).

Figure 9 shows the single/multiple cases of GP with different pathological types. Among single cases, the proportion of patients with inflammatory polyps was 6.3%; adenomatous polyps accounted for 2.0%; chronic inflammation accounted for 2.0%; inflammatory fibrous polyps accounted for 1.1%; fundus gland polyps accounted for 22.4%; and hyperplastic polyps accounted for 19.3%. Among multiple cases, the proportion of patients with inflammatory polyps was 2.4%; adenomatous polyps accounted for 0.5%; chronic inflammation accounted for 0.7%; inflammatory fibrous polyps accounted for 0.4%; basal gland polyps accounted for 25.7%; and hyperplastic polyps accounted for 17.2%. Differences of different pathological types between single and multiple GPs were remarkable (*P* < 0.05). Moreover, there were more types of adenomatous polyps and inflammatory polyps in single polyps. In multiple polyps, there were more types of fundus gland polyps and hyperplastic polyps (*P* < 0.05).

Figure 10 shows the HP infection of different pathological types. The proportion of HP-positive patients with inflammatory polyps was 6.7%; adenomatous polyps accounted for 1.7%; chronic inflammation accounted for 2.3%; inflammatory fibrous polyps accounted for 1.3%; fundus gland polyps accounted for 36.8%; and hyperplastic polyps accounted for 26.4%. Different pathological types were compared in pairs, and there was no substantial difference (*P* > 0.05).

## 4. Discussion

Based on the SIFT algorithm, the SIFT feature vector was merged with the feature vector of the image area, and a new feature vector was constructed for feature point matching, to complete the medical image registration and stitching. CT imaging technology based on IMA was proposed to process medical CT images. The results showed that not only it can effectively realize image stitching but also the stitched image quality is superior to the traditional SIFT method. It was consistent with the research results of Xia et al. [12].

GP is usually found in the upper gastrointestinal endoscopy, usually asymptomatic and accidentally diagnosed, most of which are present in epithelial GP. There was a total of 588 GP patients, including 154 males and 434 females, with a male-to-female ratio of 1 : 2.818. The number of females was relatively larger, and the prevalence rate was high. There was obvious difference in prevalence between genders (*P* < 0.01). GP patients were the most distributed in the 60–69 age group (216 people, 36.73%), indicating that more attention should be paid to the symptoms of women and elderly patients. Olmez et al. [6] found that, of 192 GP patients, 51 were males (26.6%) and 151 were females (73.4%). The average age of the patients was 61.9 ± 13.3 (14–90) years. Hyperplastic polyps, adenomatous polyps, and fundus gland polyps accounted for 88%, 2.6%, and 1.6%, respectively. The size of polyps in 70% of patients was ≤1 cm. The most common sites for polyps were the antrum and gastric body. The results were consistent with those of this work. GP was found in all parts of the stomach cavity, and the incidence of gastric fundus and gastric body was higher, accounting for 28.62% and 36.85%, respectively. Fundus gland polyps and hyperplastic polyps accounted for a relatively large number of 48.25% and 36.62%, respectively. Proliferative polyps were mostly found in the stomach body and antrum, and fundus gland polyps were mostly found in the stomach body and fundus. The polyp sites between the two groups were very evident (*P* < 0.05). It was consistent with the results of Chen et al. [13] who reported that the common pathological types of GP were fundus glands (52.27%) and hyperplastic polyps (34.74%). Sánchez-Montes et al. [14] found that 62% of 827 GP patients were female, and 53.9% of patients had multiple polyps. The most common location was the fundus of the stomach, and 83.3% had GP smaller than 1 cm. Prado-Núñez et al. [15] found that 74.3% of female had an average age of 61.5 years, most of the lesions were located in the stomach and antrum, 74.29% of polyps were less than 1 cm in diameter, and 83.64% of them are sessile. Most GPs were proliferative gastric cancer (76.4%), followed by fundus gland polyps (17.5%) and gastric adenomas (6.1%). The above results were similar to those of this study, which found that the comparison of different pathological types was not obvious regarding HP infection condition (*P* > 0.05). Studies suggested that HP infection can cause mucosal inflammatory hardening, thus leading to the formation of polyps. The occurrence and development of these lesions may be affected by environmental factors such as HP infection [16].

## 5. Conclusion

IMA was applied to process CT images, so as to analyze the pathological characteristics of GP patients. It was found that IMA-based CT imaging technology not only can effectively realize image stitching but also was superior to traditional SIFT method in terms of stitched image quality. Ultrasound images based on image mosaic algorithm clearly showed that hyperplastic polyps were mostly found in gastric antrum, and gastric fundus polyps were mostly found in gastric fundus. However, there are still some shortcomings in this study. For example, the number of samples is limited, and the basic information of patients included is limited. In the future, it can consider increasing the number of samples and conducting the discussion of patients' occupation, BMI, and other medical history. In short, the results of this study can provide a reference for GP's imaging diagnosis and follow-up treatment research.

## Figures and Tables

**Figure 1:** Flow chart of IMA.

**Figure 2:** Performance comparison of different algorithms. (a) AMBE value. (b) *H* value.

**Figure 3:** CT image of some patients. (a) Male, 61 years old, abdominal distension, vomiting, and gastric fundus gland polyp. (b) Female, 63 years old, abdominal distension and hyperplastic polyp. (c) Female, 59 years old, hyperplastic gastric antrum polyp, and round mass.

**Figure 4:** Gender composition of patients.

**Figure 5:** Age distribution of patients.

**Figure 6:** Pathological distributions of patients regarding their smoking and drinking conditions (1: inflammatory polyp; 2: adenomatous polyps; 3: chronic inflammation; 4: inflammatory fibrous polyps; 5: fundus gland polyps; 6: hyperplastic polyps) (^*∗*^indicated that relative to fundus gland polyps, the differences were evident, *P* < 0.05).

**Figure 7:** Distribution of clinical symptoms of patients (1: abdominal discomfort; 2: retrosternal discomfort; 3: weight loss; 4: nausea and vomiting; 5: abdominal pain; 6: abdominal distension; 7: sour regurgitation; 8: heartburn).

**Figure 8:** Distribution of patients with different pathological types (1: inflammatory polyp; 2: adenomatous polyp; 3: chronic inflammation; 4: inflammatory fibrous polyp; 5: fundus gland polyp; 6: hyperplastic polyp).

**Figure 9:** Single/multiple GPs of different pathological types (1: inflammatory polyp; 2: adenomatous polyp; 3: chronic inflammation; 4: inflammatory fibrous polyp; 5: fundus gland polyp; 6: hyperplastic polyp) (^*∗*^indicated that, in contrast to single cases, *P* < 0.05).

**Figure 10:** HP infection of different pathological types (1: inflammatory polyp; 2: adenomatous polyp; 3: chronic inflammation; 4: inflammatory fibrous polyp; 5: fundus gland polyp; 6: hyperplastic polyp).

**Table 1:** GP size and Yamada typing results.

		Fundus gland polyps	Hyperplastic polyps	Inflammatory polyps	Adenomatous polyps	Chronic polyps	Inflammatory fibrous polyps	Total
Polyp size (cm)	≤0.5	41.8	19.9	6.9	0.3	2	0.3	71.2
	0.6–1	6.9	9.4	2.2	1	0.8	0	20.3
	1.1–2	0.5	3.8	0.3	0.4	0.2	0.5	5.7
	≥2	0	2.7	0	0.1	0	0	2.8
	Total	49.2	35.8	9.4	1.8	3	0.8	100

Yamada type	I	12.3	5.9	1.9	0	0.6	0.4	21.1^*∗*#^
	II	36.2	27.4	7	2	1.8	0.9	75.3^*∗*#^
	III	0.2	2.6	0	0	0.3	0.2	3.3
	IV	0.1	0.2	0	0	0	0	0.3
	Total	48.8	36.1	2.6	2	2.7	1.5	100

Note: ^*∗*^and ^#^were statistically different from III and IV, respectively (*P* < 0.05).

**Table 2:** Distribution characteristics of GP parts (*N* (%)).

	Inflammatory polyps	Chronic polyps	Inflammatory fibrous polyps	Adenomatous polyps	Fundus gland polyps	Hyperplastic polyps	Total
Cardia	2.98	0.57	0	0.23	0.78	2.13	6.69
Pylorus	0	0.22	0	0	0	0.58	0.8
Body sinus junction	0.26	0.17	0	0	1.28	1.39	3.1
Substrate junction	0.18	0	0	0	1.12	0.98	2.28
Stomach body	1.38	0.76	0.26	0.53	19.56	14.36	36.85
Fundus of stomach	0.48	0	0	0.23	24.33	3.58^*∗*^	28.62
Gastric antrum	3.02	1.06	0.9	1.26	1.78	12.61^*∗*^	20.63
Angle of stomach	0.59	0	0.22	0	0	0.22	1.03
Total	8.89	2.78	1.38	2.25	48.85	35.85	100

Note: ^*∗*^showed statistical difference compared with the basal gland polyp (*P* < 0.05).

## Data Availability

The data used to support the findings of this study are available from the corresponding author upon request.
